The article "Assessment of Pattern of Abdominal Injury over a Two-Year Period at St Paul's Hospital Millenium Medical College and AaBET Hospital, Addis Ababa, Ethiopia: A Retrospective Study" was published in 2022. Journal: Emerg Med Int.

# Assessment of Pattern of Abdominal Injury over a Two-Year Period at St Paul's Hospital Millenium Medical College and AaBET Hospital, Addis Ababa, Ethiopia: A Retrospective Study

**DOI:** 10.1155/2022/3036876

**Published:** 2022-09-27

**Authors:** Kassaye Demeke Altaye, Ayalew Zewdie Tadesse, Mahteme Bekele Muleta, Woldesenbet Wagenew Dode

**Affiliations:** ^1^Department of Emergency Medicine and Critical Care, University of Gondar College of Health Sciences, Gondar, Ethiopia; ^2^Department of Emergency Medicine and Critical Care, St Paul's Hospital Millennium Medical College, Addis Ababa, Ethiopia; ^3^Department of Surgery, St Paul's Hospital Millennium Medical College, Addis Ababa, Ethiopia

## Abstract

**Background:**

Globally, injury continues to be an important cause of morbidity and mortality both in developed and developing countries. Abdominal injuries are among the major causes of trauma admissions. This study aimed to assess patterns of abdominal injury at AaBET and St. Paul's Hospital Millennium Medical College.

**Methods:**

A cross-sectional study was done on all adult patients who sustained abdominal injuries presented to the emergency department and managed at AaBET and St. Paul's Hospital Millennium Medical College over a two-year period from January 2018 to December 2019.

**Results:**

A total of 165 abdominal injured patients presented during the study period. Among those patients, 140 (84.8%) were male, with a male-to-female ratio of 5.61. The mean age of patients was 29.3 years. 85 (51.5%) of the patients sustained penetrating injuries. 53 (32.1%) patients sustained road traffic accidents, 47 (32.1%) had stab injuries, and 34 (20.6%) had gunshots. Thirty-four (20.6%) of the patients were managed conservatively and 79.4% (*n* = 131) were managed surgically. The commonest complications found were shock (*n* = 20 (12.1%)), peritonitis (*n* = 18(10.9%)), HAP (*n* = 9 (5.5%)), and surgical site infection (*n* = 4 (2.4%)).The mortality rate was 3.6% (*n* = 6), of which 4 (67%) had the penetrating mechanism of injury.

**Conclusion:**

Abdominal trauma predominantly affects the male and economically productive age. The three main causes of abdominal injuries in this study were road traffic accidents, stab injuries, and gunshots, which require increased public awareness of the need to prevent road traffic accidents and to handle weapons and sharp items properly.

## 1. Background

According to the World Health Organization's (WHO) global burden of injury estimate ranks injury is one of the top ten leading causes of death, with an estimated 5 million deaths annually, among which men in Africa have the highest injury-related mortality rates in the world [1]. Trauma is the second largest cause of illness, accounting for 16% of the global disease burden, and it is the highest between the ages of 15 and 45 years. According to WHO, low- and middle-income countries account for more than 90% of all injuries. Africa, mainly the Sub-Saharan region, contributes 21% of these [2].

The article "Assessment of Pattern of Abdominal Injury over a Two-Year Period at St Paul's Hospital Millenium Medical College and AaBET Hospital, Addis Ababa, Ethiopia: A Retrospective Study" was published in 2022. Journal: Emerg Med Int.

The abdomen is vulnerable to injury since there is minimal bony protection for underlying organs [3]. The etiological spectrum and mechanism of injury of abdominal trauma, which have been reported in the literature, vary from one part of the world to another, partly because of variations in infrastructure, civil violence, wars, and crime [4]. Abdominal trauma poses a diagnostic challenge to general surgeons and professionals practicing in resource-limited countries [5].

The management of patients with abdominal trauma has several important elements: adequate prehospital care; rapid transport to a specialized Centre; complex in-hospital care; and rehabilitation. In recent years, many abdominal injuries, especially those involving solid organs are managed nonoperatively. This has been made possible by the invention of imaging techniques like ultrasonography, computerized tomography (CT) scanning, and magnetic resonance imaging (MRI), which show the site and extent of the injury [6–8].

This study aimed to assess the pattern of abdominal injuries at St Paul's Hospital Millennium Medical College (SPHMMC) and Addis Ababa Burn, Emergency and Trauma (AaBET) hospital, Addis Ababa, Ethiopia.

## 2. Methodology

This hospital-based cross-sectional study was done at SPHMMC and AaBET hospitals from January 2018 to December 2019. SPHMMC is one of the tertiary referral hospitals in Addis Ababa, Ethiopia, established in 1968. The hospital serves around 15,000 emergency visits a year and has around 700 inpatient beds. AaBET Hospital is an affiliate of SPHMMC in Addis Ababa, Ethiopia, established in 2015 for quality improvement to improve emergency, burn, and trauma care. The hospital provides emergency, critical care, general surgery, neurosurgery, and orthopedic service.

In this study, we included all patients clinically diagnosed to have an abdominal injury who presented to SPHHMC/AaBET Hospital from January 2018 to December 2019. Patients who died before diagnosis and patients treated at other hospitals and referred for other reasons were excluded.

### 2.1. Operational Definition

Blunt abdominal injury: is defined as damage to the abdomen and/or abdominal organs secondary to impact with a blunt (not penetrating) object or surface.

Penetrating abdominal injuries: are defined as injuries to the abdomen and/or abdominal organs secondary to a foreign body penetrating the abdomen and dissipating energy into the organs and the surrounding area.

The article "Assessment of Pattern of Abdominal Injury over a Two-Year Period at St Paul's Hospital Millenium Medical College and AaBET Hospital, Addis Ababa, Ethiopia: A Retrospective Study" was published in 2022. Journal: Emerg Med Int.

Revised Trauma Score (RTS): is one of the common scores used to quantify the severity of trauma injuries based on GCS, blood pressure, and respiratory rate.

Multisystem injury: when there are injuries to more than 2 body system injury.

Combined surgery: More than two procedures done intraoperatively.

### 2.2. Data Collection

Data were collected from the trauma registry and patient files using a pretested structured questionnaire filled out by two trained data collectors. The questionnaire was categorized into sociodemographics (age, sex, residency, and address), clinical profile (triage, v/s, type of injury, associated injury), management, and outcome (management, complications, disposition, and mortality). The completeness of the data were checked by the principal investigator.

### 2.3. Data Analysis

The collected data was entered and analyzed using the statistical software SPSS version 25.0. Descriptive statistics were employed and summarized in the form of proportions and frequency tables for categorical variables. Continuous variables were summarized using mean and interquartile ranges (IQR).

Ethical clearance was obtained from SPHMMC IRB.

## 3. Results

### 3.1. Sociodemographics

A total of 9693 trauma patients were evaluated at AaBET and SPHMMC hospitals in the study period, of which one hundred sixty-five (1.7%) patients had abdominal trauma. One hundred forty (84.8%) were males, with a male-to-female ratio of 5.6 : 1. The mean age was 29.4 years with an SD of 11.7.99 (60.0%) were from the Oromia region, 55 (30.9%) from Addis Ababa (Table 1).

### 3.2. Clinical Profile

Seventy-eight (47.3%) patients were initially triaged as orange. Eighty-five (51.5%) patients had the penetrating injuries. Fifty-three (32.1%) patients sustained RTA while 47 (28.5%) had stab injuries. Twenty-three patients (15.3%) had associated polytrauma while 20(13.3%) had associated chest injury (Table 2).

### 3.3. Management and Complications

131 (79.4%) patients were managed surgically, while 34 (20.6%) patients were managed conservatively. 76 (46.1%) of patients were transfused. Of operated patients, 38 (23%) patients had spleen injury, of this 30 (78.9%) had a blunt abdominal injury.

Shock (*n* = 20 (12.1%)) followed by peritonitis (*n* = 18 (10.9%)) were the most complications following surgery (Table 3).

Fifty (38.1%) of the patients had combined surgical procedure, followed by 34 (25.9%) of the patients had repair of hollow and solid organ laceration/perforation (Table 4).

### 3.4. Disposition from ED

From the Emergency Department, 134 (81.2%) were admitted to the surgical ward, 16 (9.7%) were discharged from the ED, 14 (8.05% were admitted to ICU, and 1 (0.6%) was transferred to another hospital.

The article "Assessment of Pattern of Abdominal Injury over a Two-Year Period at St Paul's Hospital Millenium Medical College and AaBET Hospital, Addis Ababa, Ethiopia: A Retrospective Study" was published in 2022. Journal: Emerg Med Int.

The mortality rate was 3.6% (*n* = 6), of which 4 (67%) had the penetrating mechanism of injury.

## 4. Discussion

Abdominal trauma continues to be a major cause of trauma admission all over the world and contributes significantly to high morbidity and mortality [3]. The majority of the patients in this study are in their 2^nd^ to 4^th^ decade of life, which represents the economically productive age group in Ethiopia, and this finding conforms to observations made by a study from Tanzania [9]. Even though we did not assess use of alcohol and drugs, other studies suggest high use in this age group [10].

In this study, more males (75.3%) were affected than females, with a male-to-female ratio of 5.6 : 1, and this is also comparable with other studies done in our setting [11]. This might be due to male's engagement in high-risk activities; and male are bread earners of most households and are probably more involved in activities that predispose them to get injured in the process of trying to earn a living and the young age group being the mobile population more involved in recreational activities like other studies [12].

In our study, penetrating trauma was the leading mechanism of abdominal injury which is in agreement with other studies [13–18]. Contrary to the above studies other researchers showed blunt injury is more common than penetrating [9, 19]. This variation could be because of variations in the mechanism of trauma [20].

Road traffic accidents, stab injuries, and gunshots were the main causes of abdominal trauma, similar to other studies [11, 13, 21]. This requires national policies and implementations to decrease road traffic accidents, stab injuries, and gunshots.

Polytrauma, followed by chest and pelvic trauma, were the three main associated traumas in patients with abdominal trauma in this study. Higher associated polytrauma and a chest injury in abdominal trauma are linked with higher mortality in different studies [22].

The operative rate in the current study was 79.4%, a figure which is comparable with that Kenyatta National Hospital (70%) [18]. In operated patients, the spleen was found to be the most commonly injured intraabdominal organ in blunt abdominal injuries, whereas the colon and small bowel were injured most in penetrating abdominal injuries like in other studies [23].

If there is no apparent evidence for laparotomy, nonoperative therapy of abdominal trauma differs depending on the kind of injury (blunt or penetrating), hemodynamic condition, FAST findings, and CT scan results. Follow-up of abdominal conditions, serial hematocrit determination, ultrasound/CT if required, and admission to the observation area are all part of the nonoperative care of blunt abdominal injuries in hemodynamically stable patients without bowel injury or significant solid organ injury. Nonoperative treatment for penetrating abdominal injuries is determined by hemodynamic stability, the lack of peritonitis, and the trajectory of the stabbing or shooting damage [24–27].

The article "Assessment of Pattern of Abdominal Injury over a Two-Year Period at St Paul's Hospital Millenium Medical College and AaBET Hospital, Addis Ababa, Ethiopia: A Retrospective Study" was published in 2022. Journal: Emerg Med Int.

The mortality rate of this study was relatively better than Kenyatta National Hospital (12.5%) [18], and operated patients' mortality in the previous same-site study (8.5%) [11]. This could be because of study inclusion criteria, injury severity differences, patient management, or clinical course.

## 5. Conclusion

Abdominal trauma predominantly affects the male and economically productive age. Road traffic accidents, stab injuries, and gunshots were the leading causes of abdominal injuries. The research urges the development of correct handling and usage of weapons and sharp items as well as the raising of public awareness about preventing traffic accidents.

## Figures and Tables

**Table 1:** Sociodemographic characteristics of patients with abdominal injuries presented to AaBET and SPHMMC emergency departments from January 2018 to December 2019.

Variable	Variable	Frequency	Percentage
*Sex*	Male	140	84.8%
	Female	25	15.2%

*Age*	0–20	36	21.8%
	21–40	109	66%
	41–60	17	10.3%
	>60	3	1.8
	Total	150	100.0

*Residency*	Urban	127	77%
	Rural	38	23%

*Region*	Oromia	99	60%
	Addis Ababa	51	30.9%
	Amhara	7	4.2%
	Afar	3	1.8%
	Debub	3	1.8%
	Benishangul	1	0.6%
	Tigray	1	0.6%

**Table 2:** Clinical profile of abdominal trauma patients presented to SPHMMC/AaBET, Addis Ababa, Ethiopia from January 2018 to December 2019.

Variable		Frequency	Percentage
*Triage site*	Red	40	24.2
	Orange	78	47.3
	Yellow-green	47	28.5

*RTS * ^*∗*^ * -score*	<or = 4	1	0.6
	>4	164	99.4

*E-FAST^*∗*^*	Positive	105	63.6
	Negative	44	26.5
	Indeterminate	3	1.8
	Not done	13	7.9

*Types of abdominal injury*	Blunt	80	48.5
	Penetrating	85	51.5

*Causes of abdominal injury*	RTA	53	32.1
	Stab	47	28.5
	Gunshot	34	20.6
	Falls	13	7.9
	Assaults	7	4.2
	Stick	5	3.0
	Stone	2	1.2
	Horn	3	1.8
	Blast	1	0.6

*Associated injury*	Multitrauma	23	15.3
	Chest	20	13.3
	Pelvic	7	4.7
	Extremity	6	4.0
	Head	4	2.7
	Spine	1	0.7
	None	89	59.3

^*∗*^RTS, Revised Trauma Score; ^*∗*^E-FAST.

**Table 3:** Management and complications of patients with abdominal injury presented to SPHHMC/AaBET hospitals, Addis Ababa, Ethiopia from January 2018 to December 2019.

Variable	Variable	Blunt	Penetrating	Total	%
Management	Conservative	26	8	34	20.6%
	Surgical	54	77	131	79.4%
*Transfusion*	Yes	46	30	76	46.1%
	No	34	55	89	53.9%
*Organ injured of operated patients*	*Spleen*	30	8	38	23%
	*Colon*	8	22	30	18.2%
	*Small bowel*	7	20	27	16.4%
	*Liver*	13	10	23	13.9%
	*Diaphragm*	6	11	17	10.3%
	*Stomach*	3	12	15	9.1%
	*Retroperitoneal hematoma*	5	6	11	6.7
	*Kidney*	6	3	9	5.5%
	*Omentum*	0	4	4	2.4%
	*Pancreas*	2	0	2	1.2%
	*Mesentery*	1	1	2	1.2%
	*Rectum*	0	2	2	1.2%
*Complication*	*Shock*	11	9	20	12.1%
	*Peritonitis*	8	10	18	10.9%
	*HAP*	6	3	7	4.3%
	*Post op intra abdominal collection*	4	1	5	3.0%
	*SSI*	2	2	4	2.4%
	*ARDS*	2	0	2	1.2%
	*Wound dehiscence*	0	1	1	0.6%
	*Aspiration pneumonia*	0	1	1	0.6%
	*UTI*	0	2	1	0.6%
	*Intussusceptions*	1	0	1	0.0%

The article "Assessment of Pattern of Abdominal Injury over a Two-Year Period at St Paul's Hospital Millenium Medical College and AaBET Hospital, Addis Ababa, Ethiopia: A Retrospective Study" was published in 2022. Journal: Emerg Med Int.

**Table 4:** Surgical procedures done for abdominal trauma patients presented to SPHHMC/AaBET hospitals, Addis Ababa, Ethiopia from January 2018 to December 2019.

Type of surgery	Frequency	Percentage
Combined surgery	50	38.1
Repair	34	25.9
Splenectomy	27	20.6
Repair and end to end anastomosis	22	16.7
Colostomy	12	9.1
Negative laparotomy	11	8.3
Lavage	6	4.5
FB removal	1	0.7

## Data Availability

The data used to support the findings of this study are available from the corresponding author upon request.

## Abbreviations

AaBET: Addis Ababa Burn, Emergency and Trauma
ARDS: Acute respiratory distress syndrome
CT: Computerized tomography
ED: Emergency department
E-FAST: Extended focused assessment with sonography for trauma
FB: Foreign body
HAP: Hospital-acquired pneumonia
ICU: Intensive care unit
IRB: Institutional review board
MRI: Magnetic resonance imaging
RTA: Road traffic accidents
SPHMMC: St. Paul's Hospital Millennium Medical College
SSI: Surgical site infection
UTI: Urinary tract infection.
